The article "Compound phenotype of osteogenesis imperfecta and Ehlers–Danlos syndrome caused by combined mutations in COL1A1 and COL5A1" was published in 2019. Journal: Biosci Rep.

# Compound phenotype of osteogenesis imperfecta and Ehlers–Danlos syndrome caused by combined mutations in *COL1A1* and *COL5A1*

**DOI:** 10.1042/BSR20181409

**Published:** 2019-07-26

**Authors:** Zejia Lin, Jican Zeng, Xinjia Wang

**Affiliations:** The Second Hospital, Shantou University Medical College, Shantou, Guangdong 515041, China

**Keywords:** COL1A1, COL5A1, Ehlers-Danlos syndrome, Osteogenesis imperfecta, Whole exome sequencing

## Abstract

Osteogenesis imperfecta (OI) is an inherited connective tissue disorder with a broad clinical spectrum that can overlap with Ehlers–Danlos syndrome (EDS). To date, patients with both OI and EDS have rarely been reported. In the present study, we investigated a family with four members, one healthy individual, one displaying OI only, and two displaying the compound phenotype of OI and EDS, and identified the pathogenic mutations. Whole exome sequencing was applied to the proband and her brother. To verify that the mutations were responsible for the pathogenesis, conventional Sanger sequencing was performed for all members of the family. We identified a known *COL1A1* (encoding collagen type I α 1 chain) mutation (c.2010delT, p.Gly671Alafs*95) in all three patients (the proband, her brother, and her mother) in this family, but also a novel heterozygous *COL5A1* (encoding collagen type V α 1 chain) mutation (c.5335A>G, p.N1779D) in the region encoding the C-terminal propeptide domain in the proband and her mother, who both had the compound phenotype of OI and EDS. The results of the present study suggested that the proband and her mother presented with the compound OI–EDS phenotype caused by pathogenic mutations in *COL5A1* and *COL1A1*.

## Introduction

Osteogenesis imperfecta (OI), or brittle bone disease, is a clinically and genetically heterogeneous disorder that mainly results in osteopenia, bone fragility, blue sclerae, dentinogenesis imperfecta, and hearing loss [1]. OI can be classified into types I–IV, and approximately 85–90% of individuals with OI have a mutation in either collagen type I α 1 chain (*COL1A1*) or collagen type I α 2 chain (*COL1A2*). Type I collagen is the most abundant protein in bone, skin, and the tendon extracellular matrix [2]. The OI Mutation Consortium, an international collaboration of many laboratories that identify OI mutations, has found that 80% of *COL1A1/COL1A2* mutations give rise to substitution of glycine residues in the type I collagen chain, and the remaining 20% of mutations result in abnormalities of mRNA splicing [3]. Mutations in the gene coding type I procollagen produce a range of disorders, including autosomal dominant OI and the rare arthrochalasis subtype of Ehlers–Danlos syndrome (EDS) [4–6]. EDS is a connective tissue disorder that is characterized by abnormal wound healing, easy bruising, atrophic scarring, and joint hypermobility [7]. Classic-type EDS (cEDS) occurs because of a *COL5A1/2* (encoding collagen type V α 1 or 2 chain) mutation and is inherited in an autosomal dominant manner. It is estimated that approximately 50% of patients with cEDS harbor a *COL5A1* or *COL5A2* mutation [7].

The article "Compound phenotype of osteogenesis imperfecta and Ehlers–Danlos syndrome caused by combined mutations in COL1A1 and COL5A1" was published in 2019. Journal: Biosci Rep.

In the present study, we report a rare family presenting with a compound phenotype of OI and EDS, such as multiple fractures, blue sclerae, atrophic scarring, easy bruising, and joint hypermobility. To understand the basis of the disorder, provide a theoretical foundation for genetic counseling, and to determine whether patients simultaneously harbor pathogenic mutations in genes associated with OI and EDS, whole exome sequencing was performed. We identified a *COL1A1* mutation known to be responsible for OI, and a novel C-propeptide domain mutation in *COL5A1*. To the best of our knowledge, this is the first report of patients with compound phenotypes of OI and EDS that harbor both *COL1A1* and *COL5A1* mutations.

## Materials and methods

The study was approved by the Ethics Committee of the Second Hospital, Shantou University Medical College. Written informed consent was obtained from each individual for their DNA to be used for research purposes.

### DNA extraction

DNA extraction was performed using a QIAamp DNA Mini Kit (Cat. No. 51104, Qiagen, Hilden, Germany) according to the manufacturer’s protocol. Genomic DNA was obtained from peripheral blood samples from the family members (Figure 1), including the proband (III-1), her brother (III-2), and their parents (II-1, II-2).

**Figure 1:** Family pedigree The diagonal lines indicate individuals with OI. The gray shading indicates individuals with OI and EDS. / = deceased.

### Whole exome sequencing

#### Library preparation and sequencing

Whole exome sequencing was performed for the two affected children (III-1, III-2) at the Beijing Novogene Bioinformatics Technology Co., Ltd (Beijing, China). Exome sequences were enriched using an Agilent liquid capture system (Agilent SureSelect Human All Exon V6; Agilent Technologies, Santa Clara, CA, U.S.A.) according to the manufacturer’s protocol. First, genomic DNA was randomly fragmented to an average size of 180–280 bp using a Covaris S220 sonicator (Covaris, Brighton, U.K.). Second, the DNA fragments were end-repaired and phosphorylated, followed by A-tailing and ligation at the 3′ ends with paired-end adaptors (Illumina, San Diego, CA, U.S.A.) with a single ‘T’ base overhang, and purified using AMPure SPRI beads from Agencourt (Azincourt, France). Then, the size distribution and concentration of the libraries were determined using an Agilent 2100 Bioanalyzer and qualified by using real-time PCR. The DNA libraries were then sequenced on an IlluminaHiSeq 4000 sequencer for paired-end 150 bp reads at Beijing Novogene Bioinformatics Technology Co., Ltd. The raw data were saved as a FASTQ (fq) format file.

The article "Compound phenotype of osteogenesis imperfecta and Ehlers–Danlos syndrome caused by combined mutations in COL1A1 and COL5A1" was published in 2019. Journal: Biosci Rep.

#### Selection of valid sequencing data

Initially, reads with adapter contamination were filtered out. Then, reads that contained more than 10% uncertain nucleotides and paired reads with single reads of low quality (Phred-like quality score (Q score) <5) were also discarded.

#### Sequencing data mapping to reference sequences and variant calling

The valid sequencing data were mapped to the reference human genome (UCSC hg19) using Burrows–Wheeler Aligner (BWA) software (version 0.7.8; https://sourceforge.net/p/bio-bwa/mailman/message/32169236/). Subsequently, Samtools software 1.0 (also from Sourceforge) was used to sort the BAM files. Picard (http://broadinstitute.github.io/picard) was then employed to identify and delete duplicates. Finally, Samtool smpileup and BCF tools were used to perform variant calling and identify single nucleotide polymorphisms (SNPs) and indels, which were stored as a variant call format (VCF) file.

#### Functional annotation and variant filter

ANNOVAR (http://annovar.openbioinformatics.org/en/latest/) was used to annotate the VCF file. The variant position, variant type, conservation prediction, and other information were obtained at this step using a variety of databases, such as dbSNP, 1000 Genome, ExAC, CADD, and HGMD. Gene transcript annotation databases, such as Consensus CDS, RefSeq, Ensembl, and UCSC, were also applied for annotation to identify amino acid alterations. Variants were filtered with a Minor Allele Frequency (MAF) > 0.1% in the 1000 Genomes databases (1000 Genomes Project Consortium). Then, synonymous single nucleotide variants (SNVs) were discarded and the retained nonsynonymous SNVs were submitted to PolyPhen-2, SIFT, MutationTaster, and CADD for functional prediction. A nonsynonymous SNV was retained if at least two out of the four software programs showed it to be ‘not benign’. Finally, we focused on genes known to be associated with OI and EDS.

#### Sanger sequencing of candidate variants

To confirm the candidate variants identified by whole exome sequencing, Sanger sequencing was performed for all members of the family displaying complicated phenotypes of OI and EDS. Primers were designed by using Premier Primer 5 software (PREMIER Biosoft International, Palo Alto, CA, U.S.A.). We used genomic DNA to amplify the region of the respective variant using Takara ExTaq® Hot Start Version (RR006A; Takara, Shiga, Japan). The Beijing Genomics Institute performed the purification of the PCR-amplified DNA and Sanger sequencing (using an ABI 3730XL sequencer).

The article "Compound phenotype of osteogenesis imperfecta and Ehlers–Danlos syndrome caused by combined mutations in COL1A1 and COL5A1" was published in 2019. Journal: Biosci Rep.

### Evolutionary conservation analysis

To evaluate the evolutionary conservation of the site of the novel *COL5A1* mutation, the protein sequences of *COL5A1* from eight animal species, including human, rhesus, mouse, elephant, opossum, chicken, *Xenopus laevis*, and zebrafish, were aligned using ClustalW embedded in MEGA7 (https://www.megasoftware.net/).

## Results

### Clinical characteristics of a Chinese family with OI

This OI family had two patients with a compound OI and EDS phenotype, a patient with only OI, and a healthy individual (Figure 1). In this family, the female proband (III-1), who was 18 years old, appeared to be healthy before the age of 12 years. Thereafter, fractures of long bones occurred three times, and her knee ligament ruptured when she was involved in a car accident at 17 years old. She also presented with blue sclerae, atrophic scarring, joint hypermobility, prominent ears, and easy bruising (Table 1 and Figure 2).

**Table 1:** Clinical features of all members of the proband’s family

		Family		
	Proband (III1)	III2	II1	II2
Age (years)	18	14	40	42
OI phenotype				
Multiple fractures	+	+	+	-
Dentinogenesis	-	-	-	-
Imperfect				
Blue sclerae	+	+	+	-
Hearing loss	-	-	-	-
EDS phenotype				
Joint hypermobility	+	-	+	-
Joint laxity	+	-	+	-
Easy bruising	+	-	+	-
Atrophic scarring	+	-	+	-
Ligament rupture	+	-	-	-
Other symptoms				
Prominent ears	+	+	+	-

**Figure 2:** Radiographic images, magnetic resonance imaging, and photographs of the findings in proband III-1 Radiographic images: (**A**) right tibia fracture, (**B**) right femoral fracture. (**C,D**) Magnetic resonance imaging (MRI) of the posterior cruciate ligament rupture in the right knee-joint. Photographs of joint hypermobility (**E,F**), atrophic scarring (**G**).

Similarly, the proband’s mother (II-1), 40 years old, not only presented with multiple fractures of long bones and blue sclerae, but also suffered from easy bruising after minor trauma, atrophic scarring, joint hypermobility, joint laxity, and prominent ears (Table 1). The proband’s brother (III-2) was 14 years old, and showed multiple fractures of long bones and blue sclerae, but did not have easy bruising, atrophic scarring, joint hypermobility, or joint laxity (Table 1). In this family, the proband’s father (II-2), 42 years old, was healthy (i.e., presented no symptoms of OI or EDS); all patients had normal mental development and normal hearing (Table 1).

The article "Compound phenotype of osteogenesis imperfecta and Ehlers–Danlos syndrome caused by combined mutations in COL1A1 and COL5A1" was published in 2019. Journal: Biosci Rep.

### Identification of mutations

To identify the causative mutations of OI in the family, whole exome sequencing was performed on proband (III-1) and her brother (III-2). The total raw data comprised 27.35 GB for the proband and her brother. An average of 98.2% of the reads had a Q score greater than 20, and 95.5% of the reads had a Q score greater than 30. Quality control indicated that 99.4% of the raw data were valid sequencing data. For III-1 and III-2, the average sequencing depth on target was 165.5× and 129.4×, respectively, and the fractions of the target covering a depth of at least 10× were 99.5 and 99.6%, respectively.

In this family, we not only found a heterozygous mutation (c.2010delT, p.Gly671Alafs*95) in *COL1A1* in III-1 and III-2, but also observed a novel heterozygous mutation of *COL5A1* (c.5335A>G). To validate the results of whole exome sequencing, Sanger sequencing was performed on the entire family. The *COL1A1* mutation (c.2010delT) was identified in all patients (II-1, III-1, and III-2) (Figure 3A), and the *COL5A1* mutation (c.5335A>G) was only identified in the proband (III-1) and her mother (II-1) (Figure 3B). Neither mutation was found in the father (II-2) (Figure 3A,B). *COL5A1* (c.5335A>G) resulted in the substitution of an asparagine residue in the C-propeptide domain in the proband (III-1) (Figure 3C). No potential variants were found in 18 other genes (*BMP1, COL1A2, CREB3L1, CRTAP, FKBP10, IFITM5, MBTPS2, P3H1, P4HB, PLOD2, PLS3, PPIB, SERPINF1, SERPINH1, SPARC, TMEM38B, WNT1*, and *SEC24D*) associated with OI or in 10 other genes (*ADAMTS2, B3GALT6, B4GALT7, COL3A1, COL5A2, DSE, FKBP14, PLOD1, PLOD3*, and *TNXB*) associated with EDS. The *COL5A1* mutation was predicted by SIFT, Mutation Taster, CADD, and Polyphen2 to be deleterious, disease causing, damaging, and benign, respectively. This mutation was classified as uncertain significance and likely benign in ClinVar database**.** Comparison of the *COL5A1* protein sequences from related animal species indicates that this *COL5A1* mutation occurred at an evolutionarily conserved site (Figure 3D).

**Figure 3:** *COL1A1* and *COL5A1* variants, structure of the collagen type V α-chain, and evolutionary conservation of the *COL5A1* mutated site (**A**) Sequences of the genomic region mutated in *COL1A1*. The mutation in the mother (II-1), proband (III-1), and brother (III-2) are marked by black arrows. (**B**) Sequences of the mutation in *COL5A1*. The mutation in the mother (II-1) and proband (III-1) are marked by black arrows. (**C**) Structure of collagen type V α-chain: purple indicates the site of the mutation (c.5335A>G, P. N1779D) in the C-terminal propeptide. (**D**) The site of the *COL5A1* mutation is evolutionarily conserved. The mutation is marked by a red arrow.

The article "Compound phenotype of osteogenesis imperfecta and Ehlers–Danlos syndrome caused by combined mutations in COL1A1 and COL5A1" was published in 2019. Journal: Biosci Rep.

## Discussion

We characterized three patients with OI and a healthy individual from the same Chinese family. Among them, two patients had a compound OI and EDS phenotype, manifesting as multiple fractures, blue sclerae, atrophic scarring, easy bruising, and joint hypermobility. To understand cause of the phenotypic variability, we performed whole exome sequencing and identified a *COL1A1* mutation and a novel *COL5A1* mutation in the patients with the compound OI/EDS phenotype.

Type I collagen is the most abundant organic component of bone, skin, and tendon extracellular matrix [2]. To date, more than 1000 *COL1A1/2* mutations have been identified in patients with OI. OI caused by *COL1A1/2* mutations is classified into two types. The first type involves the substitution of a glycine within the Gly-x-y triplet domain of the triple helix, which can give rise to the abnormal synthesis of collagen fibrils. The second type of mutation takes the form of frameshift, nonsense, and splice-site mutations, which can result in haploinsufficiency [1,8].

In this family, the patient (proband (III-1), her mother (II-1), and her brother (III-2)) have the heterozygous *COL1A1* mutation (c.2010delT) and the *COL1A1* mutation in proband (III-1) and her brother (III-2) were inherited from their affected mother. This frameshift mutation (c.2010delT) has been reported in type I/IV OI [9,10], and is predicted to cause premature termination at codon 94 [10], which could result in haploinsufficiency. Thus, our results further support the view that the *COL1A1* mutation (c.2010delT) can result in OI.

The proband’s brother harbors only the c.2010delT *COL1A1* mutation, and only has the clinical symptoms of OI. However, the phenotypes of the proband (III-1) and her mother are different from those of her brother. Interestingly, we identified an additional heterozygous gene mutation in the region of *COL5A1* encoding the C-terminal propeptide domain, which correlates with the EDS phenotype, and the *COL5A1* mutation in proband (III-1) is inherited from her affected mother. This finding may explain why the phenotypes of proband III-1 and her mother are different from those of proband’s brother. The molecular basis of cEDS is essentially a deficiency of type V collagen, which is a quantitatively minor fibrillar collagen that is widely distributed in a variety of connective tissues [11]. The major variant of type V collagen is a heterotrimer that is composed of two pro-α1 (V) chains and a single pro-α2 (V) chain, which are encoded by the *COL5A1* and *COL5A2* genes, respectively [12,13].

The article "Compound phenotype of osteogenesis imperfecta and Ehlers–Danlos syndrome caused by combined mutations in COL1A1 and COL5A1" was published in 2019. Journal: Biosci Rep.

The *COL5A1* gene encodes the α1 chain of type V collagen, which is a minor fibrillar collagen found in ligament and tendons, as well as other tissues [14]. Mutations in the *COL5A1* C-terminal propeptide domain can cause ‘functional’ haploinsufficiency of type V collagen [15,16], either because of inefficient trafficking of the mutant protein through the endoplasmic reticulum [17] or the impaired incorporation of the mutant α1 chain into type V collagen, and is an important factor in the pathogenesis of cEDS [16,18]. The mutant α1 chain of type V collagen also plays a negative role by disrupting the interactions with other ECM components, which can be observed in patients with *COL5A1* mutations in the C-terminal propeptide domain [19].

Type I and V collagens are the two main components of ligaments. Thus, mutations in *COL1A1* and *COL5A1* are potential risk factors for ligament rupture [20], as displayed by our proband. The action of an external force could make the ligament easier to rupture. The proband experienced ligament rupture caused by trauma resulting from a car accident, not from a spontaneous rupture. In addition, the proband’s mother had no history of trauma, and had not suffered ligament rupture. The type V collagen plays a central role in collagen fibrillogenesis and co-assembles with type I collagen to form heterotypic fibrils [12,23]. Type V collagen intercalates into the core of type I collagen fibrils, where it is involved in the organization and regulation of type I collagen fibril diameter [21]. In *col5a1*^+/−^ mice, tendons have larger diameter fibrils, resulting in an irregular shape [22]. Irregularly shaped fibrils generate a diminished dynamic mechanical response of *col5a1*^+/−^ tendons [22], and *COL5A1* mutations give rise to structural tendon pathology and low tendon stiffness responsible for joint hypermobility [23]. The *COL5A1* mutation (c.5335A>G) results in a change from asparagine to aspartic acid. However, interpreting the *COL5A1* mutation as disease causing without some functional studies is a limitation of our report. Mutations described previously in the C-propeptide domain of the *COL5A1* gene have involved Cysteine residues. Cysteine residues form disulfide bonds between collagen chains and changing Cysteine to another amino acid interferes with the ability of the individual collagen molecule to assemble into a trimer [18]. The effect of a mutation involving asparagine to aspartic acid change in the C-propeptide domain of *COL5A1* has been not reported. However, the c.5335A>G mutation in *COL5A1* was predicted by SIFT, Mutation Taster and CADD, respectively, to be deleterious, disease causing and damaging, indicating that this mutation could be potentially causative of disease, consistent with a role in EDS. In support of this, the site of this *COL5A1* mutation is evolutionarily conserved, suggesting that it has an important biological function. Other known and potential pathogenic variants for OI and EDS were not identified by whole exome sequencing in this family. In addition, the *COL5A1* mutation was not found in the proband’s brother, who did not display the clinical symptoms of EDS. Finally, mutations in *TNXB*, which has been associated with EDS and *COL1A1* can give rise to overlapping phenotypes of OI and EDS [24]. Therefore, we speculated that the combined mutations in *COL1A1* and the *COL5A1* C-terminal propeptide domain could result in the hybrid EDS-OI phenotype of the proband III-1 and her mother, both of whom exclusively carry the *COL5A1* (c.5335A>G) mutation within the family. Further functional studies with a larger sample size are needed to confirm the results.

The article "Compound phenotype of osteogenesis imperfecta and Ehlers–Danlos syndrome caused by combined mutations in COL1A1 and COL5A1" was published in 2019. Journal: Biosci Rep.

In conclusion, in a family with OI, we identified a *COL1A1* mutation known to be responsible for OI, and further identified a novel second mutation in the *COL5A1* C-terminal propeptide domain in patients with OI and EDS. These results suggested that a combination of *COL5A1* and *COL1A1* mutations might lead to compound phenotypes of OI and EDS. To the best of our knowledge, this is the first report showing that members of a family with both *COL1A1* and *COL5A1* mutations present with a hybrid phenotype of OI and EDS. In addition, our results support the conclusion that that *COL1A1* (c.2010delT) can result in OI. Whole exome sequencing can help us to understand the basis of diseases with compound phenotypes and provide a theoretical foundation for genetic counseling.

## Abbreviations

cEDS: classic-type EDS
COL1A1: collagen type I α 1 chain
COL1A2: collagen type I α 2 chain
COL5A1: collagen type V α 1 chain
EDS: Ehlers–Danlos syndrome
OI: osteogenesis imperfecta
SNP: single nucleotide polymorphism
SNV: single nucleotide variant
VCF: variant call format

## References

[1] MariniJ.C., ForlinoA., CabralW.A., BarnesA.M., San AntonioJ.D., MilgromS. (2007) Consortium for osteogenesis imperfecta mutations in the helical domain of type I collagen: regions rich in lethal mutations align with collagen binding sites for integrins and proteoglycans. Hum. Mutat.28, 209–22110.1002/humu.2042917078022PMC4144349

[2] ForlinoA. and MariniJ.C. (2016) Osteogenesis imperfect. Lancet16, 1657–1671, 10.1016/S0140-6736(15)00728-XPMC738488726542481

[3] GlorieuxF.H. (2008) Osteogenesis imperfecta. Best Pract. Res. Clin. Rheumatol.22, 85–100, 10.1016/j.berh.2007.12.01218328983

The article "Compound phenotype of osteogenesis imperfecta and Ehlers–Danlos syndrome caused by combined mutations in COL1A1 and COL5A1" was published in 2019. Journal: Biosci Rep.

[4] CalzavaraPintonP. and RitelliM. (2017) Delineation of Ehlers–Danlos syndrome phenotype due to the mutation (c.934C>T, p.Arg312Cys) in *COL1A1*: report on a three-generation family without cardiovascular events, and literature review. Am. J. Med. Genet.173, 524–5302810259610.1002/ajmg.a.38035

[5] ByersP.H., DuvicM., AtkinsonM., RobinowM., SmithL.T., KraneS.M. (1997) Ehlers–Danlos syndrome type VIIA and VIIB result from splice-junction mutations or genomic deletions that involve exon 6 in the *COL1A1* and *COL1A2* genes of type I collagen. Am. J. Med. Genet.72, 94–10510.1002/(SICI)1096-8628(19971003)72:1<94::AID-AJMG20>3.0.CO;2-O9295084

[6] SymoensS., SteyaertW., DemuynckL., De PaepeA., DiderichK.E., MalfaitF. (2017) Tissue-specific mosaicism for a lethal osteogenesis imperfect *COL1A1* mutation causes mild OI/EDS overlap syndrome. Am. J. Med. Genet.173, 1047–105010.1002/ajmg.a.3813528261977

[7] MalfaitF., WenstrupR.J. and De PaepeA. (2010) Clinical and genetic aspects of Ehlers-Danlos syndrome, classic type. Genet. Med.12, 597–60510.1097/GIM.0b013e3181eed41220847697

[8] RauchF., LalicL., RoughleyP. and GlorieuxF.H. (2010) Relationship between genotype and skeletal phenotype in children and adolescents with osteogenesis imperfecta. J. Bone Miner. Res.25, 1367–13741992943510.1359/jbmr.091109

[9] WardL.M., LalicL., RoughleyP.J. and GlorieuxF.H. (2001) Thirty-three novel *COL1A1* and *COL1A1* mutations in patients with osteogenesis imperfecta types I-IV. Hum. Mutat.17, 43410.1002/humu.112411317364

[10] BalasubramanianM., SobeyG.J., WagnerB.E., PeresL.C., BowenJ., BexonJ. (2016) Osteogenesisimperfecta: ultrastructural and histological findings on examination of skin revealing novel insights into genotype-phenotype correlation. Ultrastruct. Pathol.40, 71–7610.3109/01913123.2016.114025326863094

[11] HildebrandK.A., FrankC.B. and HartD.A. (2004) Gene intervention in ligament and tendon: current status, challenges, future directions. Gene Ther.11, 368–37810.1038/sj.gt.330219814724683

[12] MayerK., KennerknechtI. and SteinmannB. (2013) Clinical utility gene card for: Ehlers-Danlos syndrome types I-VII and variants - update 2012. Eur. J. Hum. Genet.21, 10.1038/ejhg.2012.16222892533PMC3533317

[13] FichardA., TilletE., DelacouxF., GarroneR. and RuggieroF. (1997) Human recombinant alpha1(V) collagen chain. Homotrimeric assembly and subsequent processing. J. Biol. Chem.272, 30083–3008710.1074/jbc.272.48.300839374485

[14] BirkD.E. (2001) Type V collagen: heterotypic type I/V collagen interactions in the regulation of fibril assembly. Micron32, 223–23710.1016/S0968-4328(00)00043-311006503

[15] De PaepeA., NuytinckL., HausserI., Anton-LamprechtI. and NaeyaertJ.M. (1997) Mutations in the *COL5A1* gene are causal in the Ehlers-Danlos syndromes I and II. Am. J. Hum. Genet.60, 547–5549042913PMC1712501

The article "Compound phenotype of osteogenesis imperfecta and Ehlers–Danlos syndrome caused by combined mutations in COL1A1 and COL5A1" was published in 2019. Journal: Biosci Rep.

[16] SymoensS., SyxD., MalfaitF., CallewaertB., De BackerJ., VanakkerO. (2012) Comprehensive molecular analysis demonstrates type V collagen mutations in over 90% of patients with classic EDS and allows to refine diagnostic criteria. Hum. Mutat.33, 1485–149310.1002/humu.2213722696272

[17] SymoensS., MalfaitF., RenardM., AndreJ., HausserI., LoeysB. (2009) *COL5A1* signal peptide mutations interfere with protein secretion and cause classic Ehlers–Danlos syndrome. Hum. Mutat.30, E395–E40310.1002/humu.2088718972565

[18] MitchellA.L., SchwarzeU., JenningsJ.F. and ByersP.H. (2009) Molecular mechanisms of classical Ehlers–Danlos syndrome (EDS). Hum. Mutat.30, 995–100210.1002/humu.2100019370768PMC3827857

[19] ZoppiN., GardellaR., De PaepeA., BarlatiS. and ColombiM. (2004) Human fibroblasts with mutations in *COL5A1* and *COL3A1* genes do not organize collagens and fibronectin in the extracellular matrix, down-regulate alpha2beta1 integrin, and recruit alphavbeta3 Instead of alpha5beta1 integrin. J. Biol. Chem.279, 18157–1816810.1074/jbc.M31260920014970208

[20] PosthumusM., SeptemberA.V., O’CuinneagainD., van der MerweW., SchwellnusM.P. and CollinsM. (2009) The *COL5A1* gene is associated with increased risk of anterior cruciate ligament ruptures in female participants. Am. J. Sports Med.37, 2234–224010.1177/036354650933826619654427

[21] NiyibiziC., KavalkovichK., YamajiT. and WooS.L. (2000) Type V collagen is increased during rabbit medial collateral ligament healing. Knee Surg. Sports Traumatol. Arthrosc.8, 281–28510.1007/s00167000013411061296

[22] JohnstonJ.M., ConnizzoB.K., ShetyeS.S., RobinsonK.A., HuegelJ., RodriguezA.B. (2017) Collagen V haploinsufficiency in a murine model of classic Ehlers-Danlos syndrome is associated with deficient structural and mechanical healing in tendons. J. Orthop. Res.35, 2707–271510.1002/jor.2357128387435PMC5632109

[23] NielsenR.H., CouppéC., JensenJ.K., OlsenM.R., HeinemeierK.M., MalfaitF. (2014) Low tendon stiffness and abnormal ultrastructure distinguish classic Ehlers-Danlos syndrome from benign joint hypermobility syndrome in patients. FASEB J.28, 4668–467610.1096/fj.14-24965625122555

[24] MackenrothL., Fischer-ZirnsakB., EgererJ., HechtJ., KallinichT., StenzelW. (2016) An overlapping phenotype of Osteogenesis Imperfecta and Ehlers-Danlos syndrome due to a heterozygous mutation in *COL1A1* and biallelic missense variants in *TNXB* identified by whole exome sequencing. Am. J. Med. Genet.170A, 1080–108510.1002/ajmg.a.3754726799614

